The article "The Potential Benefits of Nanotechnology in Treating Alzheimer's Disease" was published in 2021. Journal: Biomed Res Int.

# The Potential Benefits of Nanotechnology in Treating Alzheimer's Disease

**DOI:** 10.1155/2021/5550938

**Published:** 2021-07-04

**Authors:** Tan Sook Ling, Shanthini Chandrasegaran, Low Zhi Xuan, Tong Li Suan, Elaine Elaine, Durrgashini Visva Nathan, Yam Hok Chai, Baskaran Gunasekaran, Shamala Salvamani

**Affiliations:** ^1^Department of Biotechnology, Faculty of Applied Sciences, UCSI University, 1, Jalan Puncak Menara Gading, Taman Connaught, 56000 Kuala Lumpur, Malaysia; ^2^Division of Applied Biomedical Science and Biotechnology, School of Health Sciences, International Medical University, Bukit Jalil, 57000 Kuala Lumpur, Malaysia

## Abstract

Alzheimer's disease is a neurodegenerative disorder that is caused by the accumulation of beta-amyloid plaques in the brain. Currently, there is no definitive cure available to treat Alzheimer's disease. The available medication in the market has the ability to only slow down its progression. However, nanotechnology has shown its superiority that can be applied for medical usage and it has a great potential in the therapy of Alzheimer's disease, specifically in the disease diagnosis and providing an alternative approach to treat Alzheimer's disease. This is done by increasing the efficiency of drug delivery by penetrating and overcoming the blood-brain barrier. Having said that, there are limitations that need to be further investigated and researched in order to minimize the adverse effects and potential toxicity and to improve drug bioavailability. The recent advances in the treatment of Alzheimer's disease using nanotechnology include the regeneration of stem cells, nanomedicine, and neuroprotection. In this review, we will discuss the advancement of nanotechnology which helps in the diagnosis and treatment of neurodegenerative disorders such as Alzheimer's disease as well as its challenges.

## 1. Introduction

Alzheimer's disease (AD) is an acquired neurodegenerative disease leading to a progressive and untreatable cognitive and behavioral impairment [1–3]. The pathogenesis of AD is associated with the formation of amyloid-*β* (A*β*) plaques extracellularly and neurofibrillary tangles intracellularly [4, 5]. These induce neuronal cell death and the loss of synapse which is initiated first before progressively leading to the cognitive deficit [6, 7]. AD being known as the commonest form of dementia amongst the elderly population [8] can however present itself in two forms which are the rare early-onset dementia leading to AD (EOAD) occurring before the age of 65 and the common late-onset AD (LOAD) or known as senile dementia occurring after the age of 65 due to aging [9–11]. AD is usually the cause of plaque formations in the hippocampus of the brain that is responsible for encoding memories, as well as other parts of the cerebral cortex that is crucial for proper judgements and making decisions [1]. Besides cognitive impairment such as memory loss, the impairment in behaviors can be seen through common neuropsychiatric symptoms such as depression, agitation, delusion, and hallucinations [12].

In 2018, the estimated number of patients consisting of all ages suffering from AD in America was approximately 5.7 million, in which LOAD contributed to more than half of the estimated cases. As the size of the U.S. population that is over the age of 65 continues to increase, the number of Americans suffering from AD continues to grow and the estimated number is expected to reach 88 million patients by 2050 [13].

There are various drugs available that aim to target in treating AD; however, the most common drawback is due to the blood-brain barrier (BBB). Due to the lack of effective therapeutic medicine available to treat AD, hence only symptomatic treatment is being given to AD patients. However, in recent years, the development of nanotechnology has shown great potential in overcoming this limitation. Nanotechnology involves the modification or development of desired materials with structures sized between 1 and 100 nanometers [14]. Nanomaterials have a large surface area and its high surface to volume ratio is highly advantageous as it has significant effects on its structure. The properties of nanomaterials are lighter, stronger, faster, smaller, and more durable hence potentially making it a promising material for drug delivery especially in the case of treating cancer and AD [15]. Hence, in this review, we will discuss how nanotechnology can be used as a potential therapeutic strategy for Alzheimer's disease.

## 2. Therapy for Alzheimer's Disease

### 2.1. Drug Delivery

In order for a drug to have its maximum therapeutic effect, it is important for the drugs to retain its bioavailability, pharmacodynamics, and pharmacokinetics. Hence, the integration of a drug into or onto a polymeric and/or lipidic nanoparticle (NP) is aimed at greatly enhancing the pharmacotherapy effect of a drug (Figure 1). The use of NPs is beneficial in drug delivery process as it increases the bioavailability of a drug by improving the aqueous solubility and increases the drug half-life which in turn reduces the rate of drug clearance as well as delivering the drug to its targeted site of action [16].

As mentioned previously, the main limitation for drugs in AD treatment is due to the blood-brain barrier (BBB); hence, it is important to recognize the structure and functionality of the BBB to be able to propose different alternatives to deliver AD drugs via the nanodrug delivery system. The utilization of the binding affinity of lipid-soluble NPs towards the endothelial cells can amplify the rate of transport of a drug via endocytosis or lipophilic transcellular pathways. Besides that, the adsorptive characteristic of NPs can be advantageous as it can adsorb onto the blood capillaries of the BBB thus increasing the probability for the target drug to be transported beyond the barrier. Furthermore, the modification of NPs with specific receptors can enhance the uptake of drugs across BBB through carrier protein and receptor-mediated transcytosis [17].

Despite the ability of NPs to permeate the BBB, only about 5% drug is able to reach the brain with the existing 95% of the drug at the inexact site of action which may lead to potential systemic side effects as the conventional route of administration of drugs fails to deliver the agent to the brain accurately [18]. However, intranasal administration of drugs has been shown to facilitate the delivery of therapeutic agents directly to the central nervous system (CNS) via the olfactory and trigeminal nerves of the nasal cavity [18, 19]. In addition, intranasal administration is safe and noninvasive and the drug is able to surpass the hepatic first-pass metabolism as well as drug degradation which will increase the bioavailability of the drug [20].

### 2.2. Protein and Peptide Delivery

The delivery of AD therapeutic protein or peptide functions in the same mechanism as the delivery of AD drugs, in which the protein or peptide is encapsulated or integrated to a NP or via the attachment to polyethylene glycol (PEGylation). The principle involved in the delivery follows the nanodrug delivery system, in which the association of a protein or peptide to NPs enables the protein or peptide molecules to cross the BBB. The intranasal administration is believed to be the most ideal route of protein or peptide delivery to the target site of action. This route allows the therapeutic agent to be directly transported to the CNS without passing through the gastrointestinal tract or blood, thus safeguarding it from proteolytic degradation [21].

Based on several researches carried out on AD rat models, the delivery of proteins or peptides using NPs has conclusively proven to be a stable, effective, and safe treatment for AD. Nevertheless, this delivery system has its own set of limitations such as high cost, limited or unstable bioavailability, and some toxic effects [22].

### 2.3. Mitochondrial Targeting Treatment

Several studies have hypothesized that the mitochondria play an important role in the pathophysiology of AD. The reduction of brain metabolism or increased reactive oxygen species (ROS) causes mitochondrial dysfunction which eventually leads to the apoptosis of nerve cells in the brain thus accelerating neurodegeneration [23]. Consequently, one of the approaches that are currently being focused on the treatment of AD is by targeting the production of neuronal ROS by the mitochondria [24].

The inner mitochondrial membrane is highly selective and blocks the entry of most molecules. Some of the potential strategies include conjugating ROS scavengers to a mitochondrion penetrating short peptide sequences that has distinct physicochemical properties to transport the ROS scavengers across the inner mitochondrial membrane; encapsulating antioxidant in lipidic NP to promote antioxidant intake via micropinocytosis; and conjugation of therapeutic agents with mitochondrial signal peptide to improve the recognition of transporters for mitochondrial delivery [25].

The antioxidant NP that is used to treat AD is known as ceria (CeO_2_) NPs. It was observed in research that positively charged TPP-ceria NPs are able to localize into the mitochondria in various cell lines and at the same time scavenge mitochondrial ROS efficiently to reduce oxidative stress thus capable of suppressing neuronal death in tested mouse model [26].

The evolution of nanomedicine and mitochondrion-specific nanotechnology approaches are shown in Figure 2.

### 2.4. Gene Therapy

Gene therapy is a technique that is carried out to intracellularly deliver genetic materials to elucidate a healing effect by compensating the mutated gene such as DNA or RNA. This form of therapy is aimed at replacing or correcting the mutated gene through a single administration of the desired gene [28]. A vector is commonly used as a channel to transfer the suitable genomic materials into the targeted cell in which the gene can be expressed without resulting in toxicity [29]. Viral vectors such as adenovirus, retrovirus, and lentivirus are altered and redesigned to allow expression without being able to replicate. Having said that, there is limitation to this method including immunogenicity and toxicity due to the viruses used as vector [30].

Therefore, nonviral gene carriers are being used as vectors as they can be developed in many different forms such as cationic lipids, polymers, ceramic-based nanomaterials, and silica-based NP. The organically modified silica (ORMOSIL) NPs have the ability to condense, protect, and transport DNA plasmid within cells [31].

The anionic phosphate groups present in the plasmid DNA are electrostatically attached to the cationic amino groups of the ORMOSIL NPs [32]. The average diameter of the ORMOSIL-DNA complex should be less than 60 nm for high transfection efficiency [33]. The ORMOSIL NPs can be fluorescently labelled to confirm a successful gene transfection into the cells [34]. As they are able to precipitate in the oil-in-water microemulsion, the use of corrosive solvents and other complex purification methods can be avoided. Besides that, the presence of hydrophobic and hydrophilic groups aids ORMOSIL to act as normal micelles and reverse micelles that can be loaded with biomolecules. Moreover, the organic groups on the NPs can be modified to increase the degree of flexibility for the attachment of targeting molecules as well as enhancing its stability in aqueous systems [33].

### 2.5. Antiamyloid Therapeutics

Alzheimer's disease (AD) occurs due to excessive production of *β*-amyloid (A*β*) peptide that precipitates in the brain specifically around the neurons causing loss of synaptic terminals and neuronal impairment in the hippocampus and cerebral cortex as well diminishing the quantity of certain neurotransmitters such as acetylcholine [35–37]. A*β* is a peptide that is derived through the proteolytic cleavage of a membrane protein known as amyloid precursor protein (APP), by *β*- and *γ*-secretases [38–41]. APP is an integral transmembrane protein that can be found mainly concentrated in the synapses of neurons and astrocytes [42]. Specific inhibition of *β*- and *γ*-secretases has the ability to prevent the production of A*β*; however, these inhibitions can bring about several side effects [43].

As such, iA*β*5 peptide has been discovered as antiamyloid therapeutic agent as a new treatment against AD [44]. iA*β*5 peptide inhibits A*β* fibrillogenesis as it binds to A*β* and prevents its further assembly into amyloid fibrils. However, it was seen that the iA*β*5 peptide is unstable and can be easily degraded by proteases. Hence, to construct an iA*β*5 derivative with enhanced characteristics such as higher proteolysis endurance, stability, and solubility, polyethylene glycol (PEG) and charged sequences can be attached [45]. Nonetheless, this drug has a low BBB permeability-surface area which restricts it from reaching the brain [44].

This limitation can be overcome through a nanotechnology-based intervention that allows the drug conjugated to poly (lactic-co-glycolic acid) (PLGA) to pass through the BBB. PLGA NPs have several advantages such as an increased drug loading capacity and a versatile structure allowing surface functionalization, biocompatibility, and reduced toxicity. An increased number of ligands can be attached to the surface of the NP in order to improve its affinity towards targeted cell surface [46]. The PLGA NP surface is surrounded with antitransferrin receptor monoclonal antibody (OX26) and anti-A*β* (DE2B4) that have the ability to deliver iA*β*5 peptide in an encapsulated form [47].

## 3. The Advantages of Nanotechnology to Alzheimer's Disease

As discussed, the current available treatment for Alzheimer's disease is to lower the symptoms mainly due to the limitation of the drug to overcome the BBB. Hence, nanotechnology-based therapy has the potential to curb this limitation as there are many advantages.

### 3.1. Nanotech Immunotherapy

Immunotherapy is an emerging potential solution for the treatment of cancer. The principles and design of immunotherapy are straightforward as it firstly begins by extracting the T cells of cancer patients for *in vitro* reconstruction, allowing them to be targeted to specific cancer receptors. These modified T cells are then reintroduced into the patient resulting in tumor cells to undergo apoptosis in the blood circulation without causing any adverse reactions. However, one of the main drawbacks of immunotherapy is that it can prevent the immune system-mediated tumor elimination due to the progression of tumor malignancy followed by immune suppression of the patient. Besides that, the modified and reconstructed T cells might not be completely safe for human use. Nanotechnology or nanoparticles is a suggested alternative that has the ability to overcome these limitations and hence the increasing success rate of immunotherapy by making it safe and effective [48].

### 3.2. Safe Sterilization

Silver nanoparticles have been used extensively in the medical field such as medical devices and drug formulations. The citrate-stabilized silver NP size ranges from 20 to 80 nm can be sterilized directly via *γ*-radiation and autoclave. The silver NPs were introduced to a compound producer of hydroxy radicals, enabling the replication of the sterilization-based changes in size and morphology which inferred a free radical mechanism of action. Additionally, it was observed that the sterilized silver NPs have a likelihood of causing platelet accumulation, which is an in vitro indicator thrombogenicity, in comparison to the unsterilized silver NPs that were used as controls [49].

### 3.3. Early Disease Diagnosis Approaches

Nanotechnology has been widely studied not only for its use in disease treatment but also in medical imaging in disease diagnosis. The superparamagnetic iron oxide NPs have the ability to enhance the contrast in spectroscopy imaging. Besides that, NPs can be conjugated to specific biomarkers that enable the detection of certain tumor phenotypes via ultrasound as well as the measurement of the biomarkers [50]. Other than its role in advance medical imaging-based detection, nanotechnology serves as a high-sensitivity disease detector for early diagnostics purpose and is known for its stability and reliability in performance properties [51].

### 3.4. Biosensors

Biosensor is an instrument that detects analytes through a combination of a sensitive biological recognition, such as nucleic acids, enzyme antibodies, and a physical transducer. The results are then used for qualitative and quantitative determinations. Nanomaterials such as gold nanoparticles, graphene, carbon nanotubes, and photonic crystals are being extensively used in biosensors due to the requirement of high sensitivity and selectivity, rapid detection, and low cost [52]. Besides that, the integration of nanotechnology in biosensors has brought upon many new signal transduction advancements. The establishment of instruments and procedure to quantify and image objects at a nanoscale level has allowed the growth of biosensors interacting with minute molecules that requires to be evaluated [53].

### 3.5. Sustainability

Nanotechnology, owing to its vast potential of benefits, is widely seen as one of the enablers for sustainable development such as increasing the efficiency of many production systems. The application of nanotechnology is still not being widely used, as there are still gaps and consequences that had to be extensively studied upon [54, 55]. Thus, a reduction of interest followed the initial hype, in which an in-depth research and developmental work was carried out therefore producing new and exciting results and products each year. Engineered nanomaterials represent a new class of materials with remarkable properties, with some interesting applications being available in the market and an exponential increase in number of patents, and many more under development. There are many examples of extant and potential application of nontechnology in different scientific areas especially in medicine, pharmaceutical, and biology such as cell sorting, DNA diagnostics, kidney dialysis, tips for scanning probe microscopes, targeted drug delivery devices, purification of pharmaceuticals, lab-on-a-chip, proteomics, single-cell analysis, BioMEMS, CytoSensing, enzymes, identification of toxic compounds, cancer treatment, and biophotonics [56–58].

## 4. The Limitations of Nanotechnology

There are several consequences that were discovered in the application of nanotechnology especially in the medical field [59].

### 4.1. Solubility

The solubility of NPs may differ in certain conditions such as varying temperatures. The changes in temperature can influence the interaction between NPs and the drug [60]. This can cause certain patients to encounter different therapeutic impacts which are undesirable for medical treatments. Therefore, these aspects need to be emphasized in future research of nanotechnology in AD diagnosis or therapy to bring about favorable outcomes [61].

### 4.2. Bioavailability

The administration route of NPs may affect the bioavailability of the drug that is delivered to the body. Nasal administration route is the most practical and admissible as it is one of the most noninvasive methods to administer drugs into the human body. However, the nasal cavity has enzymes that can highly affect the bioavailability of the drug [62]. Thus, this may require increasing the dosage of the drugs when administering which can cause adverse reactions in the nasal mucosa as the nasal cavity has a limited capacity of drug concentration. Therefore, it is important to administer a low concentration of drugs via the nasal route [60]. Besides that, when introducing a high volume of low bioavailable drugs, this can cause serious respiratory effects such as chronic inflammatory responses, peribronchial inflammation, and oxidative stress [63].

### 4.3. Blood-Brain Barrier

The blood-brain barrier (BBB) plays an important function in neuronal circuits and synaptic transmission [9]. However, it remains to be an impenetrable obstacle for a large number of exogenous substances such as drugs including antibiotics, antineoplastic agents, and a variety of central nervous system- (CNS-) active drugs especially neuropeptides.

Drug delivery using NPs is one of the possibilities to transport active molecules efficiently across the BBB. This is due to ligands that are functionalized onto NPs to improve the targeted drug delivery to overcome BBB [59]. However, the efficiency of these ligand-modified NPs needs to be evaluated as it still requires a long blood-residency time to be able to pass through the BBB and hit their target system [64].

### 4.4. Toxicity

Despite numerous benefits in the application of NPs, many of its components such as nucleic acids, antibody fragments, peptides, and proteins can function as antigens consequently resulting in increased immunotoxicity [65].

Although acute toxicity caused by NPs can be identified through clinical experiment, the potential chronic toxicity due to long-term exposure and accumulation of NPs should be considered too. Currently, there are no experimental studies tested on living organisms regarding the chronic toxicity of NPs to determine the toxicity and adverse effects of NPs [66]. Meanwhile, consuming high amount of nanocarriers containing surfactants and cosurfactants due to low encapsulation efficacy and loading capacity of NPs can cause serious adverse effects [61]. Certain NPs that have been administered into the body cannot be easily removed by various clearance systems. This may cause the NPs to accumulate within the brain system causing to cytotoxicity. Long-term accumulation of NPs in the brain may lead to brain injuries [67].

The sink effect of NP-mediated initiation, the frequency, and intervals between injections is one of the limitations that should be considered as well. An excessive amount of dose may cause adverse effects, which in turn initiates an immunogenic response causing the alteration of NP pharmacokinetics and diminishing its efficacy. Besides that, neurotoxicity caused by NPs may be due to its physicochemical properties such as size, shape, and surface area. These factors could potentially modulate or interfere with the transport of hemostatic mediators [59]. The size of NPs may increase the possibility of aggregation which can interfere and block the blood flow that may result in undesirable reactions in the lungs, heart, and other microinfarctions.

Although nanotechnology-based approaches have shown immense therapeutic potential, it is still in its early stage. The safety and chronic effects of NPs should be investigated further to ensure it is clinically safe and effective for the treatment of human diseases [68].

### 4.5. Cost

The production of NPs is an expensive and complex process, which needs specific ingredients, instruments, and optimal conditions, especially multifunctional NPs which can be used for both preventive and therapeutic purposes [66]. Therefore, further experimental studies should emphasize on reducing the cost/benefit ratio in the application of nanotechnology in the clinical setting as it will be applied in medical healthcare to patients.

## 5. Recent Advances in Neurology Using Nanotechnology

The applications of nanotechnology in neurological therapy involve cellular biology. There are diverse therapeutic options available for neurological disorders even for incurable Alzheimer's disease and Parkinson's disease [69]. Since there is an increase in scientific researches and research funding, the future explorations of nanotechnology in neurological disorders seem very promising. The prospects of nanoneurotechnology mainly focus on regenerative medicines. Besides that, stem cell research is an essential aspect in nanoneurotechnology. Neurodegenerative disorders are mostly provoked by ceased blood supply to tissues and reactive oxygen species. Hence, the current progression of treating neurodegenerative diseases involves inhibiting these conditions.

### 5.1. Nanoparticles in Stem Cell Regeneration

Nanomaterials are functional biological elements that exist in a nanometer range. This ensures a better interaction for the elements with the biological system. The fundamental principle of nanoneuromedicine is that the NPs enhance tissue regeneration without stimulating an immune response and warding off infections [70]. A few of the prominent usage of NPs in stem cell research includes magnetic NPs in the isolation and assortment of stem cells. Quantum dots are also used in molecular imaging and tracing of stem cells. The regulation of stem cell proliferation and differentiation can also be controlled by using NPs [71].

Organ failures remain as one of the most dreaded medical issues. Scaffolds are an important aspect of tissue engineering. Natural scaffolds are obtained through a process of decellularization while retaining the original composition of the extracellular matrix to allow recellularization using induced pluripotent stem cells, which can refurbish the functionality of organs. Stem cells maintain and generate tissues in the body and go through selective differentiation to become specialized cells. This enables stem cells to be integrated with NPs for improved cell proliferation and differentiation. Nanomaterials can also enhance the optimal control of microenvironment conditions of transplant cells. The harvested stem cells can be developed into 3-dimensional organoids. Brain studies are always hindered by limitations due to the usage of postmortem tissue [72]. This venture can pave the way for future functional studies of the human brain.

Regeneration of stem cells has to be continuously monitored and evaluated to ensure its functional and structural accuracy. Nanoparticles can also be used in confocal imaging to evaluate the bioengineered tissue. Further developments in this field have brought upon the evolution of a new branch of research which is nanotoxicology. This is because the toxicity of nanomaterials needs to be verified before the application of clinical trials [72].

### 5.2. Nanomedicine

Currently, theranostics is a new method that is being used to treat neurodegenerative disorders. Theranostics involves the application of both diagnostic and therapeutic nanomedicine. Recent advances in nanomedicine mainly focus on drug targeting. Reduction of tumor volume can be achieved by using magnetism where carmustine-integrated NPs are conducted within the brain tumor. Antiretroviral drugs are combined with theranostic NPs which applies drug targeting mechanism [69]. Hence, ligand targeting and nanoformulated particles to quantize drug dose reductions are in development.

Another type of nanomedicine that is currently being revised is liposome-encapsulated hemoglobin. These molecules are permeable to ischemic territories when there is a sudden loss of blood circulation. Therefore, inadequate blood supply in stroke models can be monitored using the liposome-encapsulated hemoglobin molecules. Cerium oxide NPs are also integrated in nanoneuromedicine to forage reactive oxygen species (ROS). CeO_2_ NPs can also be used in neuroprotection against nerve injury [69].

### 5.3. Neuroprotection

Neuroprotection is among one of the most important treatment options for neurodegenerative disorders. When there is a sudden cease of blood supply to the brain tissues, necrosis and apoptosis occur. Antioxidants are widely used as a treatment option as they have the ability to prevent cell or tissue death. However, when there are inadequate levels of antioxidants, oxidative stress occurs which causes chronic inflammation and damages to cell structure. Neuroprotection attacks oxidative stress and excitotoxicity [73]. Oxidative-mediated mutations by chemical species like superoxide (O_2_), hydroxyl (OH), and peroxide (H_2_O_2_) can cause plasma membrane lipid peroxidation and decline in mitochondrial energy production. Transporter proteins can also be inactivated [74].

Antioxidants integrated into NPs are able to eliminate free radicals that are formed in the brain. The nanomaterial that is normally used in neuroprotection is fullerene and its derivatives. Fullerenol-mediated neuroprotection inhibits free radicals besides inhibiting intracellular calcium concentrations that cause cell excitation. Currently, there are developments in the application of neuroprotection at the nanolevel. One of the examples includes the usage of carbon nanotube electrode arrays. The nanotube electrodes enhance neurorepair through nanoscaffolds. Hence, chemical substances and electrical consolidation can be equipped at the nanoscale. This allows surgeries at micro or nanolevels to be conducted for elementary axon renovation. Carbon nanotubes enable the monitoring and altering of neural activity as well as enabling synaptic plasticity [74].

## 6. Conclusion

The application of nanotechnology in the treatment of Alzheimer's disease includes the improvement of the drug, therapeutic protein, and antiamyloid delivery across the blood-brain barrier. In addition, the transport of antioxidants to the mitochondria to prevent the release of reactive oxygen species and delivery of genetic material to the cells are also the implementation of nanotechnology in Alzheimer's disease treatment. The prospects of nanotechnology in the treatment of Alzheimer's disease include advances in bioimaging and proteomics. Despite recent advancements in using nanotechnology for the treatment of Alzheimer's disease, the possibility of chronic toxicity has to be further researched for future clinical applications. Another big challenge in utilizing nanotechnology in Alzheimer's disease is the cost. The cost would be a barrier in accepting nanotechnology treatment as the common treatment for Alzheimer's disease.

## Figures and Tables

**Figure 1:** Different ways to incorporate drug into or onto a nanoparticle [1].

**Figure 2:** Evolution of nanomedicine (top) and nanotechnology approaches to mitochondrial medicine (bottom). DQA: dequalinium; TPP: triphenylphosphonium [27].
